# Antibacterial activity of *Hibiscus rosa-sinensis* L. red flower against antibiotic-resistant strains of *Helicobacter pylori* and identification of the flower constituents

**DOI:** 10.1590/1414-431X2020e10889

**Published:** 2021-05-17

**Authors:** L.T.M. Ngan, M.T. Tan, N.V.M. Hoang, D.T. Thanh, N.T.T. Linh, T.T.H. Hoa, N.T.M. Nuong, T.T. Hieu

**Affiliations:** 1 Faculty of Biology and Biotechnology, VNUHCM-University of Science, Ho Chi Minh City, Vietnam; 2 Oxford University Clinical Research Unit, Hospital for Tropical Diseases, Ho Chi Minh City, Vietnam; 3 Faculty of Applied Sciences, Ton Duc Thang University, Ho Chi Minh City, Vietnam; 4 Faculty of Chemistry, VNUHCM-University of Science, Ho Chi Minh City, Vietnam; 5 Central Laboratory for Analysis, VNUHCM-University of Science, Ho Chi Minh City, Vietnam

**Keywords:** *Hibiscus rosa-sinensis* flower, Antibacterial activity, Helicobacter pylori, Antibiotic resistance, Urease inhibition, Identified constituents

## Abstract

Utilization of plant resources for treatment of *Helicobacter pylori* infections is one of the appealing approaches as rapid emergence of antibiotic-resistant strains is occurring throughout the world. Ethanol extract and its fractions from *Hibiscus rosa-sinensis* red flower were assessed for antibacterial and urease inhibitory activities towards forty-three clinical strains and two reference strains of *H. pylori*. The ethyl acetate fraction exhibited the most potent bacteriostatic activity with minimum inhibitory concentrations (MICs) of 0.2-0.25 mg/mL and minimum bactericidal concentrations (MBCs) of 1.25-1.5 mg/mL against all test strains, including forty-three strains resistant to one to four antibiotics, azithromycin (MICs, 8-256 µg/mL), erythromycin (MICs, 8-128 µg/mL), levofloxacin (MICs, 8-256 µg/mL), and/or metronidazole (MICs, 8-256 µg/mL). The fraction had similar antibacterial activities toward these test strains suggesting the preparation and the antibiotics do not have a common mechanism of anti-*H. pylori* activity. The fraction also had stronger effects on biofilm formation, morphological conversion, and urease activity of *H. pylori* than the other fractions and the ethanol extract. These flower preparations were non-toxic to three human cell lines, and nine compounds were also isolated and identified from the ethyl acetate fraction. *In vivo* research needs to be conducted to confirm the potential usefulness of *H. rosa-sinensis* flower and its constituents for effective prevention and treatment of *H. pylori* disease.

## Introduction

*Helicobacter pylori*, a microaerobic, Gram‐negative, and spiral-shaped bacterium, is known to be a major cause of gastrointestinal diseases such as chronic active gastritis, peptic ulcer, and gastric carcinoma (1). The global prevalence of *H. pylori* infection is about 51% in developing countries compared with 35% in developed countries (2). Since the infectious agent has been known to be a human carcinogenic factor, several antibiotic therapies have been prescribed to achieve high eradication rates. However, side-effects caused by the antibiotics and recurrence of the bacterial infection have made the therapies lose their effectiveness. In addition, widespread over-the-counter use of antibiotics in some developing countries has also contributed to the emergence of *H. pylori* antibiotic-resistant strains (3).

Folk medicinal plants, particularly their extracts and phytochemicals, have been perceived as relatively safe with little or no side effects and often act at multiple and novel target sites, thereby reducing the risk of resistance development (4). A number of medicinal plant preparations traditionally used for treatment of topical wounds and gastrointestinal disorders have been reported to have anti-*H. pylori* activity (5,6). Specifically, *Hibiscus rosa-sinensis* L. (Malvaceae family), a tropical evergreen shrub with red flowers, is traditionally used for the treatment of flu and cough, bronchitis, stomach pain, dysentery and diarrhea, and also for regulation of menstruation and stimulation of blood circulation (7). Aerial part extracts of the plant have been known to possess antiulcerogenic activity on gastric ulcers (8). Extracts from leaves and flowers of the plant have been proven to possess antibacterial activity (9,10). Due to the effectiveness and safety, all parts of the plant could be used for pharmacological purposes (11,12). The phytochemical constituents, pharmacological effects, and medicinal uses of the plant have been well described (13). In our previous study, the ethanol extract and ethyl acetate fraction derived from the *H. rosa-sinensis* flower were found to have antibacterial activity against *H. pylori* ATCC 43504 and four isolated compounds (naringenin, luteolin, myricetin, and protocatechuic acid) from the fraction were also proven to possess potent antibacterial properties against seven antibiotic-sensitive and -resistant strains of *H. pylori* (14).

The present study aims to report the antibacterial and urease inhibitory effects of crude ethanol extract of the *H. rosa-sinensis* red flower and its solvent-soluble fractions against forty-three clinical strains and two reference strains of *H. pylori*. In addition, isolation and structural elucidation of nine other compounds from the ethyl acetate fraction are also reported.

## Material and Methods

The study was approved by the Ethical Committee of the Vietnam National University, Ho Chi Minh City (No. 702/DHQG-KHCN).

### Instrumental analyses

^1^H and ^13^C NMR spectra were collected on a Bruker AVANCE III spectrometer (Germany) at 500 and 125 MHz, respectively, and chemical shifts are given in δ (ppm) using CDCl_3_, CD_3_OD, (CD_3_)_2_CO, or (CD_3_)_2_SO as solvent. High-resolution mass spectrometry (HRMS) analysis was performed using a Bruker MicroTOF-QII-system with an ESI-source. Melting point was determined using a Bibby Stuart Melting point SMB3 (UK). UV spectra were measured in ethanol on a T92+ Spectrophotometer (PG instrument, UK). Merck precoated silica gel plates (Kieselgel 60 F_254_, Germany) were used for analytical thin-layer chromatography (TLC). Merck preparative layer chromatography plates (PLC silica gel 60 F_254_, 2 mm thickness) and Scharlau silica gel 60 (0.06-0.2 mm) (Spain) were used for isolation and purification.

### Materials

The E test strips of six antibiotics (amoxicillin, azithromycin, erythromycin, levofloxacin, metronidazole, and tetracycline) were purchased from AB Biodisk (Sweden). Newborn bovine serum (NBS) was purchased from Hyclone (USA). Brucella broth (BB) and brain heart infusion (BHI) broth were provided by Becton, Dickinson and Company (USA). All other chemicals and reagents used in this study were of analytical grade quality and available commercially.

### Plant material and preparation of extract and fractions

The red flower petals of *H. rosa*-*sinensis* were collected in Binh Chanh district, Ho Chi Minh city, Vietnam (10°43'21.7"N, 106°40'06.1"E) in July 2019. The species was identified by T.T. Hieu at Plant Biotechnology Laboratory, Department of Plant Biotechnology and Biotransformation, Faculty of Biology and Biotechnology, VNUHCM-University of Science, Ho Chi Minh City. A voucher specimen was deposited in the herbarium of the Department under the code HRS1001.

The flower ethanol (EtOH) extract and three solvent-soluble fractions (hexane, ethyl acetate (EtOAc), and water fractions) were obtained as previously described (14). Briefly, the air-dried petals (9.5 kg) were pulverized and extracted 3 times with absolute ethanol to yield 1352 g of the EtOH extract, subsequently partitioned with hexane, EtOAc, and water by liquid fractionation to obtain 164 g hexane, 34 g EtOAc, and 1154 g water fractions. The extract and the fractions were subsequently tested against the forty-three clinical and two reference strains of *H. pylori*.

### Bacterial strains and culture conditions

The two reference strains ATCC 43504 and ATCC 51932 and forty-three clinical strains of *H. pylori* were obtained in 2017 from the Microbiology Lab at OUCRU (Oxford University Clinical Research Unit, Vietnam). All bacterial strains were stored in BHI broth with 25% glycerol in a liquid nitrogen container and were cultured on Brucella agar supplemented with 10% NBS at 37°C for 3 days in a microaerophilic jar using Oxoid CampyGen gas packs (Thermo Scientific, UK).

### Human cell lines and cultures

HeLa cells (ATCC CCL2, cervix carcinoma cell line), Jurkat cells (ATCC TIB-152, blood cancer cell line), and MCF7 (ATCC HTB-22, human breast cancer cell line) were provided from the American Type Culture Collection (USA). HeLa, Jurkat, and MCF7 cells used were between passages 4 and 20. These cell lines were cultured in Eagle's minimal essential medium (EMEM) supplemented with 10% fetal bovine serum (FBS), 2 mM L-glutamine, 20 mM HEPES, 0.025 μg/mL amphotericin B, 100 IU/mL penicillin, and 100 μg/mL streptomycin, at 37°C and 5% CO_2_ (14).

### Microbiological assay

Minimum inhibitory concentrations (MICs) of the six antibiotics were determined by the E test method according to the manufacturer's instructions. Different antibiotics (amoxicillin, azithromycin, erythromycin, levofloxacin, metronidazole, and tetracycline) served as positive controls. MICs, minimum bactericidal concentrations (MBCs), and time-killing of the extract and fractions towards all the bacterial strains were determined using broth microdilution assay.

For MICs, serial dilutions of concentrations (0.1 to 20 mg/mL) of the extract and fractions were performed in 0.05 mL of 10% NBS-supplemented Brucella broth in sterile 96-well plates (15). The final concentration of DMSO in all assays was 2.5% or less. Subsequently, 0.05 mL of bacterial suspension (∼5×10^6^ CFU/mL) of each strain from cultures on Brucella agar was added to each well. The plates were then incubated at 37°C in microaerophilic jars and shaken at 50 rpm for 48 h. MICs are defined as the lowest concentrations that visibly inhibited bacterial growth using resazurin as an indicator. Negative controls contained the DMSO solution.

MBC values of the test materials were identified following the MIC assays and carried out in 24-well plates with Brucella agar medium (6). An amount of 0.01 mL of each well that retained the blue color of the indicator was taken and dropped onto the agar medium. The agar plates were incubated in microaerophilic jars at 37°C for 72 h. The lowest concentrations, which exhibited no growth on the subculture, were determined as MBC values.

The time-killing assay was performed in sterile 96-well plates with the test compounds at concentrations of 1-6 times the MIC. Bacterial viability was measured after 0-48 h by a plate colony count technique as described previously (15). A control without the test compounds was also performed.

### Biofilm formation inhibitory assay

Biofilm inhibition assay was performed in 96-well plates using crystal violet assay with the most active fraction at subMICs against *H. pylori* ATCC 43504 biofilm formation 48 h post-treatment as reported previously (14). Blank and background wells, which contained DMSO and the fraction, respectively, without bacterial suspension, were similarly prepared. After two days, staining with crystal violet was performed, and the biofilm formation was determined by measuring absorbance on a Microlisa Plus microplate reader (Micro Lab Instruments, India) at a wavelength of 595 nm.

### Effect on morphology of *H. pylori*

*H. pylori* ATCC 43504 was cultured in Brucella broth with or without the extract or fractions at concentrations of 0.75 and 1.5 mg/mL under microaerophilic conditions for 24 and 48 h. The bacterial suspension (15 μL) was evenly spread and fixed on slides and then stained with 0.3% methylene blue solution. The proportion of coccoid *vs* spiral-shaped bacteria was determined using a EuromexBioBlue Lab microscope equipped with a Euromex camera (The Netherlands). Counts of 200 bacteria from each slide were done as reported previously (14).

### Cytotoxicity assay

The cytotoxicity of the EtOH extract and fractions to HeLa, Jurkat, and MCF7 cells was evaluated using a sulforhodamine (SRB) assay described previously (14). In brief, cells were seeded onto 96-well plates at a density of 5×10^3^ cells/well (HeLa), 5×10^4^ cells/well (Jurkat), and 10^4^ cells/well (MCF7) for 24 h. The culture medium was then removed from the wells and replaced with a medium containing various concentrations of the extract and fractions (0−1 mg/mL) in DMSO. After incubation for 48 h, the cells were washed once with phosphate-buffered saline (PBS), fixed with cold trichloroacetic acid solution (50% w/v) for 20 min, and stained with 0.2% SRB for 20 min. After gently washing five times with acetic acid solution (1%), the protein-bound dye was solubilized in 10 mM Tris base solution. Absorbance was read at 492 nm by the microplate reader. Camptothecin (Calbiochem, Germany) was used as a positive control.

### Inhibition of urease *in vitro*

Inhibition of *H. pylori* ATCC 43504 urease was determined by measuring ammonia production in 96-well plates using the salicylate-hypochlorite method with minor modification as described previously (14). In brief, the assay mixtures containing 0.25 μg of urease crude (0.04 urease units) in 0.1 mL of the EDTA-sodium phosphate buffer (pH 7.3) and the extract and fractions at different concentrations (0-5 mg/mL) were preincubated at 37°C for 90 min with rotation at 50 rpm. An amount of 0.05 mL of urea solution (10 mM) in the sodium phosphate buffer was added to each well, and the plates were incubated for 30 min. Blank and background wells were similarly prepared but with inactive urease by heating at 100°C for 30 min. Then, stop solutions including 0.035 mL of solution A (146% Na salicylate + 0.1% sodium nitroprusside) and 0.065 mL of solution B (1.78% NaOH + 11.57% Na citrate + 0.54% NaOCl) were added in sequence. The ammonia released by the urease activity was quantified by measuring the absorbance on the microplate reader at 625 nm. The protein content was determined using a Bradford protein assay kit (Biorad, USA). BSA was used as a protein standard. Thiourea served as a standard reference inhibitor. One unit of urease is defined as the amount of enzyme that releases 1 μM NH_3_ per minute, at 37°C, pH=7.3. Each treatment was performed in triplicate and repeated three times in independent experiments.

### Isolation of major compounds in the active fraction

Due to being the most active fraction against the test *H. pylori* strains, the EtOAc fraction (30 g) was subjected to silica gel column chromatography and eluted with a gradient of hexane and EtOAc (100:0-0:100 by volume) described previously (14). In the present study, sub-fractions with similar *R*_f_ values on TLC plates were pooled together, evaporated to dryness at 42°C, and 40 sub-fractions were obtained. Repetitive silica gel column chromatography of the sub-fractions E_2_ (219.4 mg), E_8_ (1370 mg), E_11_ (2180 mg), E_12_ (725.7 mg), E_14_ (1560 mg), E_21_ (56.5 mg), and E_36_ (425.3 mg) followed or not by plate chromatography resulted in nine compounds. The scheme of isolation of these compounds is presented in Figure S1.

### Statistical analyses

MIC and MBC values of each test sample were results of at least three independent experiments. Antibacterial activity of the extract and fractions with MIC values <0.1, 0.1-0.62, >0.62-1.25, >1.25-2.5, and >2.5 mg/mL were defined as extremely high, high, moderate, low, and no growth inhibition, respectively (16). Cytotoxicity to human cell lines and urease inhibition activity are reported as CC_50_ (50% cytotoxic concentration) and IC_50_ (concentration of half-maximal urease inhibition), respectively, and determined using GraphPad Prism 5 software program (USA). The CC_50_ and IC_50_ values of the treatments were considered to be significantly different if their 95% confidence intervals did not overlap. The Bonferroni method was used to test for multiple comparisons among the treatments. The percentage of biofilm inhibition (%) was calculated as follows: 100 - 100 × (OD_treatment_ - OD_background_) / (OD_control_ - OD_blank_).

## Results

### Antibiotic resistance of *H. pylori* clinical strains

The antibacterial activity of six common antibiotics toward forty-three *H. pylori* clinical isolates is shown in Figure 1 with MIC breakpoints for these test antibiotics (17 [Bibr B18]–19). All the strains showed resistance to 1-4 test antibiotics. Four strains (9.3%) were resistant to four antibiotics (azithromycin, erythromycin, levofloxacin, and metronidazole) with MICs of 8-256 µg/mL. Sixteen strains (37.2%) were resistant to three antibiotics (azithromycin, erythromycin, and metronidazole) with MICs of 8-256 µg/mL. Thirteen strains (30.2%) were resistant to two antibiotics (five strains to erythromycin and metronidazole with MICs of 8-128 µg/mL, four strains to levofloxacin and metronidazole with MICs of 64-256 µg/mL, three strains to azithromycin and erythromycin with MICs of 16-256 µg/mL, and one strain to azithromycin and metronidazole with MICs of 64-256 µg/mL). Ten strains (23.3%) were resistant to a single antibiotic (eight strains to metronidazole with MICs of 32-64 µg/mL and two strains to levofloxacin with MICs of 256 µg/mL). No strains showed resistance to amoxicillin and tetracycline. The reference strain ATCC 51932 was sensitive to all antibiotics, whereas strain ATCC 43504 showed resistance to metronidazole with a MIC of 32 µg/mL.

**Figure 1:** Antibiotic minimum inhibitory concentration (MIC) distribution for forty-three clinical strains of *H. pylori* using the E test method. MIC breakpoints for azithromycin (AZM >1), erythromycin (ERY >0.5), levofloxacin (LEV >1), metronidazole (MTZ >8), tetracycline >1, and amoxicillin >0.5 μg/mL (refs. 17-19).

### Growth inhibitory and bactericidal activities of *H. rosa-sinensis* flower

The growth inhibitory and bactericidal activities of the extract and fractions toward the two reference strains and forty-three clinical strains are presented in Figure 2. Based on MIC values, EtOAc fraction had the highest level of growth-inhibitory activity (0.2-0.25 mg/mL), followed by the hexane fraction (moderate inhibition, 0.75-1.0 mg/mL), and the EtOH extract (low inhibition, 1.25-1.75 mg/mL). The water fraction showed very weak growth inhibitory activity.

**Figure 2:** Minimum inhibitory concentrations (MIC) and minimum bactericidal concentrations (MBC, within parentheses) of *H. rosa-sinensis* ethanol extract (EtOH ext.) and three fractions (fr.) (Hexane fr., ethyl acetate (EtOAc) fr., and Water fr.) for forty-three clinical and two reference strains of *H. pylori* using broth dilution bioassay.

Based on MBC values, the EtOAc fraction exerted the highest bactericidal activity (1.25-1.5 mg/mL), and the EtOH extract and hexane fraction did not show a significant difference in bactericidal activity (5.0-7.5 mg/mL). Noticeably, the EtOH extract and fractions were of similar growth-inhibiting activity and toxicity towards both antibiotic-susceptible and -resistant strains, although its concentrations were lower than those of the test antibiotics. The EtOAc fraction exhibited the most potency against all forty-three clinical strains of *H. pylori* resistant to 1-4 test antibiotics, and two reference strains, ATCC 43504 resistant to metronidazole and ATCC 51932 susceptible to all the six test antibiotics.

The time course of bactericidal activity of EtOAc fraction at various concentrations of 1 (0.25 mg/mL), 2 (0.5 mg/mL), 4 (1 mg/mL), 5 (1.25 mg/mL), and 6 (1.5 mg/mL) times the MIC toward *H. pylori* ATCC 43504 was likewise investigated and is reported in Figure 3. The results indicated that the viable count of the bacteria was reduced in a dose-dependent manner. Treatment of *H. pylori* with EtOAc fraction at the six and five times MIC reduced the viability of *H. pylori* by ∼6.1 log_10_ and 3.7 log_10_ at 24 and 12 h, respectively; at the four times and twice MIC resulted in ∼4.1 log_10_ and ∼2.2 log_10_ reduction at 36 and 18 h, respectively. The EtOAc fraction completely killed all the bacteria 36 h post-treatment at MBC (six times MIC). This indicated that the EtOAc fraction exhibited bacteriostatic activity toward all test *H. pylori* strains rather than bactericidal effect. Bactericidal activity of a plant preparation significantly depends on type of the extract and its components, concentration, and exposure time, as well as density of test bacterial strains.

**Figure 3:** Time-course bactericidal activity of ethyl acetate (EtOAc) fraction at different concentrations ranging from minimum inhibitory concentration (MIC=0.25 mg/mL) to minimum bactericidal concentration (MBC=1.5 mg/mL) toward *H. pylori* ATCC 43504. Data are reported as means±SE.

### Anti-biofilm formation activity

Our results of antibiofilm formation showed that EtOAc fraction at subMICs inhibited biofilm formation of *H. pylori* ATCC 43504 (Figure 4). The EtOH extract and the other two fractions did not exhibit an antibiofilm effect on the strain at all test concentrations. At concentration of 1/2 × MIC (0.125 mg/mL), 1/4 × MIC, and 1/8 × MIC, EtOAc fraction produced significant antibiofilm activity and reduced biofilm formation by 79.3, 56.4, and 44.8%, respectively (P<0.05), while at 1/16 MIC and 1/32 MIC, the fraction showed weak antibiofilm activity with no significant difference (P>0.05).

**Figure 4:** Effect of ethyl acetate (EtOAc) fraction at concentrations of subminimum inhibitory concentrations (MICs) on *H. pylori* ATCC 43504 biofilm formation 48 h post-treatment. Data are reported as means±SD.

### Effect on morphology of *H. pylori*

The proportion of coccoid versus spiral form of *H. pylori* ATCC 43504 was recorded at 0.75 and 1.5 mg/mL of the EtOH extract and fractions after 24 or 48 h treatment (Figure 5). Effect of concentration (F=1484.86; df=8, 45; P<0.0001) and exposure time (F=1092.21; df=1, 45; P<0.0001) on conversion of *H. pylori* to the coccoid form was significant. The concentration by exposure interaction was also significant (F=215.56; df=8, 45; P<0.0001). The EtOAc fraction caused considerable conversion to the coccoid forms (91 *vs* 18% at 1.5 and 0.75 mg/mL after 48 h of treatment). The hexane fraction caused higher conversion to the coccoid forms than the EtOH extract at 1.5 mg/mL (40.1 and 32.2%, respectively, P<0.001), while the hexane fraction and EtOH extract at 0.75 mg/mL did not produce a significant difference in the coccoid conversion (P>0.05). The water fraction caused the lowest conversion (11.4% at 1.5 mg/mL), and the proportion of conversion caused by the water fraction at 0.75 mg/mL was not significantly different from that of the control group (P>0.05).

**Figure 5:** Effect of *H. rosa-sinensis* flower ethanol extract (EtOH ext.), and its fractions (Hexane fr., ethyl acetate (EtOAc) fr., and Water fr.) at concentrations of 0.75 and 1.5 mg/mL on *H. pylori* ATCC 43504 morphology 24 and 48 h post-treatment. Data are reported as means±SD.

### Cytotoxicity

In order to determine the selectivity of the anti-*H. pylori* activity, the cytotoxic effects of the red flower preparations were examined (Table 1). The EtOH extract, hexane, EtOAc, and water fractions displayed no significant cytotoxicity with CC_50_ >1, 0.646−0.878, 0.339−0.445, and >1 mg/mL, respectively, towards HeLa, Jurkat, and MRF7 cell lines, compared with that of the positive control camptothecin with CC_50_ of 0.005−0.81 µg/mL (P<0.001).

**Table 1:** Cytotoxic effect (50% cytotoxic concentration, CC_50_) of *H. rosa-sinensis* flower ethanol (EtOH) extract and fractions on three human cell lines.

Sample	CC_50_, mg/mL (95%CI)		
	HeLa	Jurkat	MCF7
EtOH extract	>1	>1	>1
Hexane fraction	0.878 (0.817-0.944)	0.646 (0.626-0.666)	0.801 (0.785-0.817)
EtOAc fraction	0.445 (0.421-0.471)	0.363 (0.302-0.436)	0.339 (0.314-0.366)
Water fraction	>1	>1	>1
Camptothecin (µg/mL)	0.810 (0.704-0.932)	0.005 (0.004-0.006)	0.005 (0.004-0.006)

CI: confidence interval; EtOAc: ethyl acetate.

### Urease inhibitory activity

The flower EtOH extract and fractions inhibited the activity of *H. pylori* urease (Table 2). The EtOAc fraction exhibited the highest activity (IC_50_ at 0.101 mg/mL), caused a steep dose-response curve of percentage of urease inhibition, and complete inhibition at 0.3 mg/mL, followed by the water fraction with lower urease inhibitory activity (Figure 6). The EtOH extract and hexane fraction produced weak and no inhibition to *H. pylori* urease, respectively. However, the extract and fractions showed a lower effect than the positive control thiourea (IC_50_ at 0.044 mg/mL) (Table 2).

**Figure 6:** *H. pylori* urease inhibitory activity of *H. rosa-sinensis* flower ethanol extract (EtOH ext.) and two fractions (fr.) (ethyl acetate (EtOAc) fr. and Water fr.). Data are reported as means±SD.

**Table 2:** Concentration of half-maximal inhibition (IC_50_) of *H. rosa-sinensis* flower ethanol (EtOH) extract, fractions, and thiourea on *H. pylori* ATCC 43504 urease inhibition.

Sample	Slope±SE	IC_50_, mg/mL (95%CI)
EtOH extract	2.304±0.096	2.144 (2.100-2.190)
Hexane fraction	-	-
EtOAc fraction	2.203±0.039	0.101 (0.100-0.107)
Water fraction	1.875±0.064	0.431 (0.415-0.447)
Thiourea	1.861±0.107	0.044 (0.042-0.047)

CI: confidence interval; -: no inhibition; EtOAc: ethyl acetate.

### Identification of major compounds in EtOAc fraction derived from *H. rosa-sinensis* flower

Nine compounds from the active EtOAc fraction were obtained and identified based on melting points and spectral data such as ESI-HRMS, ^1^H-NMR, ^13^C-NMR, 2D ^1^H-^13^C HSQC, and 2D ^1^H-^13^C HMBC. These nine compounds isolated and identified in this study can be found in several plant species, and three compounds (taraxerol acetate (20), p-hydroxybenzoic acid (21), and quercetin (21)) were previously identified in *H. rosa-sinensis*. The remaining six compounds are being reported here for the first time in *H. rosa-sinensis* red flower. The structure of these identified compounds (Figure 7) were determined and further compared with the reported literature, and are in agreement with taraxerol acetate (compound 1) (C_32_H_52_O_2_, ESI-HRMS, *m*/*z* 469.4032 [M + H]^+^) (20), 5-hydroxy-7,4'-dimethoxyflavone (compound 2) (C_17_H_14_O_5_, ESI-HRMS, *m*/*z* 299.0963 [M + H]^+^) (22), velutin (compound 3) (C_17_H_14_O_6_, ESI-HRMS, *m*/*z* 315.0850 [M + H]^+^) (23), guaifenesin (compound 4) (C_10_H_14_O_4_, ESI-HRMS, *m*/*z* 221.0818 [M + Na]^+^) (24), trans-p-coumaric acid (compound 5) (C_9_H_8_O_3_, ESI-HRMS, *m*/*z* 163.0356 [M - H]^-^) (25), p-hydroxybenzoic acid (compound 6) (C_7_H_6_O_3_, ESI-HRMS, *m*/*z* 137.0219 [M - H]^-^), 5-hydroxymethylfurfural (compound 7) (C_6_H_6_O_3_), quercetin (compound 8) (C_15_H_10_O_7_, ESI-HRMS, *m*/*z* 303.0499 [M + H]^+^) (25), and fumaric acid (compound 9) (C_4_H_4_O_4_, ESI-HRMS, *m*/*z* 115.0029 [M - H]^-^). ^1^H-NMR, ^13^C-NMR, and HMBC data of the nine compounds isolated from *H. rosa-sinensis* flower are shown in Table S1 and Figure S2.

**Figure 7:** Chemical structures of nine compounds identified from ethyl acetate (EtOAc) fraction derived from *H. rosa-sinensis* flower extract.

## Discussion

In recent years, the increasing resistance of *H. pylori* to several common antibiotics has significantly decreased the efficacy of treatment and drawn global attention. Plant extracts and phytochemicals derived from medicinal plants have proven to be antibacterial agents and some of them have multiple functions and act at multiple target sites (4). Various extracts from all parts of *H. rosa-sinensis* have been reported to exhibit a wide range of beneficial effects such as hypotensive, antipyretic, anti-inflammatory, anticancer, antioxidant, antidiabetic, and antibacterial activities (8,10,13). Flower extracts of *H. rosa-sinensis* were suggested as an alternative source of antibacterial agent against human pathogens (10) and possess stronger antibacterial activity than that of the leaf against some clinical bacterial isolates, such as *Staphylococcus aureus*, *Proteus vulgaris*, *Pseudomonas aeruginosa*, and *Citrobacter* sp. (9). Methanol and hexane extracts of the flower have strong antigrowth activities against *Bacillus subtilis* and *Escherichia coli*, while ethanol extract shows strong inhibition against *Salmonella* spp. (10). In a study of medicinal plants traditionally used for gastrointestinal disorders, leaf and stem extracts from a white flower variety of *H. rosa-sinensis* exhibit moderate and low activity against metronidazole-resistant clinical isolates of *H. pylori*, respectively (5). In the present study, EtOH extract and fractions from the red flower of *H. rosa-sinensis* were proven to have antibacterial activities against both antibiotic-susceptible and -resistant strains of *H. pylori*, although its concentrations were lower than those of the test antibiotics. The EtOAc fraction exhibited the most potency against all forty-three clinical strains of *H. pylori* resistant to 1-4 test antibiotics, and two reference strains ATCC 43504 resistant to metronidazole and ATCC 51932 susceptible to all the six test antibiotics.

Numerous extracts from medicinal plants also possess antibacterial activity against antibiotic-resistant strains of *H. pylori*. Methanol extract from young stems of *Terminalia spinosa* shows strong antibacterial activity toward 12 strains of *H. pylori* (26). Natural almond skin polyphenol-rich extract has an inhibitory effect against two clarithromycin-resistant strains of *H. pylori* (27). Hexane and chloroform fractions from leaves of *Magnolia sieboldii* display strong growth inhibition to the strain ATCC 43504 (28). Ethanol extracts of *Ampelopsis cantoniensis* and *Cleistocalyx operculatus* display similar anti-*H. pylori* activity against two antibiotic-resistant clinical isolates (6). In the present study, the EtOAc fraction of *H. rosa-sinensis* flower significantly reduced the viability of *H. pylori* ATCC 43504 at 2, 4, and 5× MIC after 12-36 h of incubation, and only completely killed the strain at 6× MIC (MBC) 36 h post-treatment. This indicated that the EtOAc fraction exhibited bacteriostatic activity toward all test *H. pylori* strains rather than bactericidal effect. Bactericidal activity of a plant preparation significantly depends on the type of the extract and its components, concentration, and exposure time, as well as density of test bacterial strains. In our previous study, four compounds (naringenin, luteolin, myricetin, and protocatechuic acid) identified from the EtOAc fraction of *H. rosa-sinensis* red flower were also found to be bacteriostatic rather than bactericidal against *H. pylori* ATCC 43504 (14).

In addition, inhibitory effects of antibacterial agents against biofilm formation play a major role in the eradication of *H. pylori* infection. Methanol extract from calyces of *H. sabdariffa* was reported to have fungistatic effect against *Candida albicans* and significantly reduces biofilm formation of six strains of fluconazole resistant *C. albicans* at subMIC (1/2 and 1/4 MIC) (29). Our present study also demonstrated that the EtOAc fraction of *H. rosa-sinensis* red flower exhibited the potential inhibitory effect on *H. pylori* biofilm formation at subMIC (1/2, 1/4, and 1/8× MIC). Moreover, morphological conversion of the *H. pylori* cells from spiral to coccoid forms caused by plant preparations is one possible mechanism affecting the survival and colonization of the bacterium on the gastric mucosa. Methyl gallate, paeonol, and 1,2,3,4,6-penta-O-galloyl-β-D-glucopyranose from the root extract of *P. lactiflora* were reported to cause 91-74% coccoid conversion at 2× MIC after 48 h of treatment (16). In the present study, the EtOAc fraction from the flower extract of *H. rosa-sinensis* caused considerable conversion to the coccoid forms (91% at MBC after 48 h of treatments).

*H. pylori* urease also plays a crucial role in colonization and pathogenesis of the pathogen in the stomach. Hence, inhibition of the enzyme activity is one of the most important strategies for the treatment of the bacterial infection. Several plant preparations have been reported to possess multiple effects toward the metabolic activities of *H. pylori*. Extracts from *Camellia sinensis* were found to inhibit the bacterial growth and the function and production of urease (30). Acetone, aqueous, and methanol extracts of *Acacia nilotica*, *Adhatoda vasica, Calotropis procera*, *Casuarina equisetifolia*, and *Fagoniaar abica* traditionally used in folk medicine for the treatment of a variety of common ailments in Pakistan were reported to have anti-urease activity (31). Epigallocatechin gallate (EGCG) from the green tea plant inhibits the urease activity and motility of *H. pylori* (32). In the present study, the EtOAc fraction derived from *H. rosa-sinensis* flower exhibited the highest activity, followed by the water fraction with lower urease inhibitory activity.

Conversion of the spiral to the coccoid forms in *H. pylori* is caused by environmental factors, antibiotics (33), and phytochemicals (16). It has been suggested that coccoid forms consist of viable but non-culturable coccoid (VBNC) and non-viable degenerative coccoid forms (34). The VBNC form has minimal metabolic activity and can survive during stress conditions such as in the presence of antibiotics, which may be one of the causes of treatment failure (35). However, potent plant preparations that act through multiple mechanisms on the bacterium and could be consumed for long-term treatment due to their safety may successfully kill the bacterium including the dormant form. In the present study, the EtOAc fraction of *H. rosa-sinensis* inhibited the growth, biofilm, and urease activities of *H. pylori*. These promising effects may contribute to combat resistance and prevent recurrence of *H. pylori*. The EtOH extract, hexane, EtOAc, and water fractions of the flower showed no significant cytotoxicity towards the three cell lines (HeLa, Jurkat, and MRF7). This suggested that their anti-*H. pylori* activities might not be due to general toxicity. Previously, *H. rosa-sinensis* plant and its chemical constituents were suggested to be utilized in pharmacological applications because extracts of the flower and the leaf were considered relatively safe (11,12).

The phytochemical constituents, pharmacological effects, and medicinal uses of *H. rosa-sinensis* have been well described and the main bioactive compounds responsible for its medicinal effects are namely flavonoids, tannins, terpenoids, saponins, and alkaloids (13). Among the identified compounds shown in Figure 7, compound 2 (5-hydroxy-7,4'-dimethoxyflavone) was active against *C. albicans* with a mechanism of action including inhibition of *C. albicans*' ergosterol synthesis, drug efflux pumps, and antioxidant enzymes (22). Compound 3 (velutin) (23), compound 5 (trans-p-coumaric acid) (36), and compound 6 (p-hydroxybenzoic acid) (37) exhibited significant dose-dependent activity against both Gram-negative and -positive pathogenic bacteria, such as *Vibrio cholera*, *Salmonella* Typhimurium, *Shigella* dysenteriae, *E. coli*, *Pseudomonas aeruginosa*, *Streptococcus pneumonia*, *S. mutans, Staphylococcus aureus*, and *Bacillus subtilis*. Compound 8 (quercetin) exhibited inhibitory effect on biofilm formation by *S. mutans* (38) and inhibited *H. pylori* urease activity (39).

Among the three flavonoids (naringenin, myricetin, and luteolin) derived from the EtOAc fraction of *H. rosa-sinensis* red flower, naringenin was reported to have the most growth-inhibiting and antibiofilm activities and induced morphological transformation of *H. pylori* (14). In our present study, the EtOAc fraction exerted lower inhibitory activity than the positive control thiourea against *H. pylori* urease. However, myricetin and luteolin were found to exhibit stronger inhibitory activity than the positive control (14). It was reported that plant flavonoids may contribute to several antimicrobial mechanisms, such as inhibition of nucleic acid synthesis (by inhibiting helicase, gyrase, and topoisomerase activity), disruption of membrane function (by inhibiting efflux pumps, porins, fatty acid synthase, and peptidoglycan synthesis), inhibition of energy metabolism, quorum sensing and biofilm formation, and thereby attenuation of the pathogenicity (40). These isolated compounds in the present study may serve as the lead compounds for development of new antipathogenic agents, a critical requirement to counteract the antibiotic-resistant bacteria.

In this work, these results demonstrated that the EtOAc fraction derived from red flower extract of *H. rosa-sinensis* was highly bacteriostatic against both antibiotic-susceptible and -resistant strains of *H. pylori* through potent effects on biofilm formation, morphological conversion, and urease activity of *H. pylori*. The results suggested that the EtOAc fraction and its isolated compounds could have great potential as new, effective, and safe agents for the prevention or treatment of *H. pylori* infection.

## Supplementary Material

Click here to view [pdf].
